The article "Neurogenerative Disease Diagnosis in Cepstral Domain Using MFCC with Deep Learning" was retracted in 2023. Reasons: signs of a paper mill; compromised peer review; unreliable results or conclusions.

# Neurogenerative Disease Diagnosis in Cepstral Domain Using MFCC with Deep Learning

**DOI:** 10.1155/2022/4364186

**Published:** 2022-04-04

**Authors:** Norah Saleh Alghamdi, Mohammed Zakariah, Vinh Truong Hoang, Mohammad Mamun Elahi

**Affiliations:** ^1^Department of Computer Sciences, College of Computer and Information Sciences, Princess Nourah Bint Abdulrahman University, P.O.Box 84428, Riyadh 11671, Saudi Arabia; ^2^Department of Computer Science, College of Computer and Information Sciences, King Saud University, P.O. Box 57168, Riyadh 21574, Saudi Arabia; ^3^Faculty of Computer Science, Ho Chi Minh City Open University, 97 Vo Van Tan, Ward Vo Thi Sau, District 3. Ho Chi Minh City: 70000, Vietnam; ^4^Department of Computer Science and Engineering, United International University, Dhaka, Bangladesh

## Abstract

Because underlying cognitive and neuromuscular activities regulate speech signals, biomarkers in the human voice can provide insight into neurological illnesses. Multiple motor and nonmotor aspects of neurologic voice disorders arise from an underlying neurologic condition such as Parkinson's disease, multiple sclerosis, myasthenia gravis, or ALS. Voice problems can be caused by disorders that affect the corticospinal system, cerebellum, basal ganglia, and upper or lower motoneurons. According to a new study, voice pathology detection technologies can successfully aid in the assessment of voice irregularities and enable the early diagnosis of voice pathology. In this paper, we offer two deep-learning-based computational models, 1-dimensional convolutional neural network (1D CNN) and 2-dimensional convolutional neural network (2D CNN), that simultaneously detect voice pathologies caused by neurological illnesses or other causes. From the German corpus Saarbruecken Voice Database (SVD), we used voice recordings of sustained vowel /a/ generated at normal pitch. The collected voice signals are padded and segmented to maintain homogeneity and increase the number of samples. Convolutional layers are applied to raw data, and MFCC features are extracted in this project. Although the 1D CNN had the maximum accuracy of 93.11% on test data, model training produced overfitting and 2D CNN, which generalized the data better and had lower train and validation loss despite having an accuracy of 84.17% on test data. Also, 2D CNN outperforms state-of-the-art studies in the field, implying that a model trained on handcrafted features is better for speech processing than a model that extracts features directly.

## 1. Introduction

Neurodegenerative diseases result in alterations in neurons and the death of neural tissues and cells over time. The incapacity of neurons to recover on their own after significant damage or degradation is the fundamental explanation for this. Neurogenerative disorders include Alzheimer's disease, Ataxia, and Parkinson's disease. However, distinguishing between illnesses, especially in the early stages, can be challenging. The multiple difficulties associated and disordered situations, such as Parkinson's [1], cause changes in voice patterns. The strained, harsh, weak, and breathy voices [2] indicate an early sign or symptom associated with a disease. So highly efficient health informatics systems would be beneficial in detecting neurogenerative disorders [3] from voice and reduce clinicians' workload [4, 5].

The research and detection of illness using speech as a biomarker is vocal pathology. Whereas most vocal fold disorders may be identified by analyzing alterations in the auditory speech signal, identifying distinct pathology situations inside of an associated multiclass clustering technique is challenging. The diagnosis of an illness at an early stage is critical, and speech signals may help with this. Voice samples are affected by many troubles such as muscle infection, residual stress, inflammation of the skin, changes to the nervous systems, and a slew of other messes situations [1]. But some of them are frequently presenting a sign of early warning among an illness, such as Parkinson's tone sounds pinched, loud, faint, or nasally due to the changed working and structure of a vocal tract [2]. Consequently, voice-based preemptive multiclass disease classification is typically a practical, simple, and widely used strategy that could lead towards a complete follow-up treatment or procedure.

A variety of other circumstances may cause vocal disorders: infections of voice tissue, weariness, climate conditions, muscle dystrophy, facial discomfort, and other symptoms [1]. Voice pathology impairs vibration regularity and voice functioning, increasing vocal noise. The familiar voice became strained, weak, and hoarse [6], affecting voice quality [7]. Voice problems comprise dysphonia, laryngitis, Reinke's edema, vocal fold nodules and polyps, vocal cord paralysis, and other vocal ailments [8, 9]. Dysphonia is a speech disorder characterized by a nodule in the vocal cords, laryngeal enlargement, or a shocking event in the vocal cords. Around 10% of the world's population is affected by this disease [10]. Another familiar voice problem is laryngitis, characterized by swelling of the vocal folds. The sickness may develop acute when viruses assault the vocal folds [9]. Reinke's edema may occur as a result of excessive stress or from immoral practices such as smoking and loud shouting. Other vocal anomalies may occur as a result of the factors mentioned above. Almost all vocal illnesses cause the voice to sound scratchy and rough. Because neurological impulses create voice, these issues may also affect brain cells [11]. Thus, negligent attitudes avoid severe circumstances that, in some instances, are not treatable by surgery and may result in horrible cancer. Early identification of vocal disorders may lessen the likelihood of severe consequences.

Existing voice pathology diagnostic technologies are biased and reliant on subjective considerations [12]. Auditory-perceptual evaluation in hospitals is an example of comprehensive interpretation, extensively used among symbolic laryngostroboscopy evaluation [13]. Numerous clinical evaluations are used to assess the rate of severity diagnosis for auditory-perceptual characteristics [14]. However, this assessment approach is parameter sensitive, time-consuming, and difficult [15]. Furthermore, these treatments include a physical examination of the patient in the clinics, which might be difficult for patients suffering from severe conditions. A kind of objective assessment involves using a computer-aided instrument to recognize and analyze speech sounds without the need for surgery. Automated detection can identify imperceptible audio to hear vocalizations [1]. These assessment procedures are not subjective, even when they do not depend on human judgment. Moreover, because the audio recordings can be viewed virtually utilizing different internet recording applications, these are easy to use. Consequently, various studies, including such [16], have developed voice recognition approaches that may be combined with such a machine learning approach to automatically detect oral pathologies in one paradigm, allowing healthy people and people with voice abnormalities to be distinguished effectively. For objective evaluation of speech pathology, many vocal pathology records have been broadly utilized in the literature. The most often used vocal pathology databases are the Saarbruecken Voice Database (SVD) [17], Arabic Voice Pathology Database (AVPD) [18], and Massachusetts Eye and Ear Infirmary Database (MEEI) [19]. Scholars often study the vowel /a/ vocalization since it is available in numerous language databases [6]. Scholars are looking into other vowel pairs [20]. The majority of research in speech diseases, for example, has limited their datasets to specific pathology sets [20].

The vast majority of studies on utilizing ML and DL to identify language illnesses have focused on binary classification, which predicts whether such a speech sample is normal or pathologic [21, 22]. For voice sickness detection, support vector machine (SVM), Gaussian mixture model (GMM), decision tree (DT), K-nearest neighbors (KNN), and other standard ML approaches have been widely used. Several deep learning methods, including artificial neural networks (ANN), convolutional neural networks (CNN), long short-term memory (LSTM)—CNN hybrid, and bidirectional LSTM, have been investigated in the past for this purpose. Previously, a variety of public voice datasets were employed for this research. For example, the MEEI, SVD, and VOICED datasets have all been utilized to discriminate between healthy and diseased voices [23]. Regrettably, most of the studies focused on only two class labels, with precision rates ranging from 70 to 94%.

This study developed and implemented a system for detecting pathological voice patterns using deep learning methods. In order to construct the most optimal classification model, two types of classifiers based on the following deep learning algorithms were investigated: 1 D CNN and 2D CNN. Both of the models were trained using the sustained vowel /a/ recording collected from the SVD database. 1D CNN was trained on raw data, and 2D CNN was trained on extracted characteristics. This work also presented a comparison of the performance of the two models.

List of contributions are the following:

- Implemented a 1D CNN model from raw audio and a 2D CNN model based on extracted MFCC features and compared their performances
- This paper utilizes sample padding and segmentation to lengthen shorter samples or split the longer samples. These methods make all the samples in the dataset to uniform duration and avoid class imbalance problems
- Determine whether raw audio signals or speech signal attributes extracted from audio are more effective at distinguishing disordered voices from healthy voices
- There is minimal feature extraction overhead because only one feature is required to successfully distinguish pathological voices
- Performance comparison of our models with other researchers' work on the same research problem

The rest of the paper is organized as follows: Section 2 describes the literature review; Section 3 discusses the details about the dataset and preprocessing techniques; Section 4 details about the methodology which consists of feature extraction, model architecture, and evaluation metrics; and Section 5 describes the results and with discussion and Section 6 with conclusions followed by a list of relevant references.

## 2. Literature Review

Artificial intelligence-based approaches have proven effective in a wide range of real-world situations [24, 25]. Machine learning algorithms have been used widely by several researchers to learn the voice manifestations of pathological states, which will reduce the difficulty of voice-based pathology diagnosis [26, 27]. A wide variety of handmade characteristics (in both the time and frequency domain representations) have been utilized to describe the signals, including entropy, energy, time, the included Mel-frequency cepstral coefficients (MFCC), cepstral domains, frequency, harmonics-to-noise ratio, and normalized noise energy [28, 29]. Those feature vectors are then loaded into a new classification algorithm [30, 31].

Disorganized speech signals are detected by [32] utilizing multitaper MFCC features and a classifier based on the Gaussian mixture model (GMM). [28] create an SVM (support vector machine) for binary pathological condition diagnosis utilizing characteristics gathered by correlation functions study on multiple frequency bands. [33] apply the ANN (artificial neural network) and SVM (support vector machine) models for classification. Aside from the fact that it is disease-specific, the majority of studies [34, 35] focuses on employing sounds of sustained vowel /a/ recorded in a clinical environment, while others [36, 37] indicate a high value with 200 recordings of sustained vowels. Several studies [28, 33, 36] have used a combination of the vowels “a,” “i,” and “u” while neglecting pathological causes, to excellent effect. In a binary classification framework, [36] generates a dataset with three different categories of speech pathology samples. While such a clinically instructive data gathering approach in the absence of a health professional may not be a practical option in a home-like situation, these techniques create a reduced binary classification job to detect just one disease-specific voice problem pattern.

As a consequence, the scientific community often overlooks numerous rare diseases. As a result of using a large-scale voice database (SVD) [14], this study can classify speakers from 71 distinct disease-specific pathology conditions, which is a relatively new and more challenging work of classification. Some of the ailments we are tackling in this project to build a multiclass classifier have never been addressed previously. Deep learning-based models have also been utilized in several recent studies to improve binary classification performance [38]. [39] propose utilizing a deep neural network (DNN) to distinguish between regular and sick classes. [40] present a convolution neural network (CNN) model using short-time Fourier transform (STFT) features for feature extraction for binary classification of voice samples. [41] use a convolutional deep belief network (CDBN) to identify pathological conditions in a binary classification framework using average and sick voice spectrograms as input. [35] apply a CNN to handle the problem of voice pathology detection. The majority of current speech-based automated depression detection techniques [42–44] depend on the relevance of auditory parameters such as pitch, intensity, jitter, shimmer, harmonic-to-noise ratio, and speech speeds to forecast a person's depressed condition. These voice quality features are linked to the idea that unhappy speakers tend to speak in an unnatural and monotonous way. Based on the recent collection of works [45–48], majority of them have implemented deep neural network models for the diagnosis of depression.

It is worth noting that the difficulty of creating a multiclass classifier capable of differentiating signals representing many disease states inside a single model has yet to be addressed. As a result, although deep learning models for voice analysis may perform better at drawing a high-level binary conclusion, the learned deep descriptors are frequently just excellent at identifying the overall qualities of input. The published study results vary significantly due to discrepancies in the databases used in the experimental investigations. The reliability attained by employing 200 records of prolonged vowel /a/ reflects a high value, according to Martínez et al. [34], which is pretty close to our study. Similar studies that did not focus on the pathological causes employed the vowels /a/, /i/, and /u/ in conjunction to achieve high accuracy. Souissi et al. [37] used a subgroup that included four categories of voice problems totaling 71 kinds to achieve high precision of 87.82% in their study. A 99.68% accuracy rate was attained by Al-Nasheri et al. [49] by testing a sample of diseases from other publicly available datasets, such as the Arabic Voice Pathology Database (AVPD) and the Massachusetts Eye and Ear Infirmary Database (MEEID) (MEEI). Another study by Muhammad et al. [36] employed a subset of three forms of vocal abnormalities and achieved a 93.20% accuracy rate.

Furthermore, they improved the accuracy to 99.98% by using a mix of speech recordings as an electroglottograph signal. Hemmerling et al. [27] used their technique to discriminate between male and female speakers and reached a high precision of 100% in the recognition problem. Hammami et al. [50] looked at how the recommended tall order statistic feature highlights produced from wavelet space may be used to discriminate between healthy and sick sounds. Traditional traits including Cruel Wavelet Esteem, Cruel Wavelet Vitality, and Cruel Wavelet Entropy were used in the experiments. These highlights attain the most significant accuracy of 99.26% during the locating phase and 100% while categorizing the data when combined with an SVM classifier. To incorporate concrete logical included values, a clinical assessment was conducted on information obtained from participants at a therapeutic institution in Tunez. The results were good, with location precision of 94.82% and classification accuracy of 94.44%, correspondingly. Fonseca et al. [51] focused on discovering coexisting laryngeal problems with the same principal phonic side effect, resulting in interclass coverage characteristics. Estimated accuracy of 95% was achieved using the proposed technique, which used SE, ZCR, and SH for extraction and DPM, particularly for arrangement. These methods were all employed to extract the data. Rueda and Krishnan's database [52] is an ongoing challenge in dysphonia voice research. Using complex deep learning algorithms without underfitting or overfitting is tricky. They invented an adaptive technique for breaking down a signal into its component pieces that uses a Fourier-based synchrosqueezing change (FSST) to expand and modify information. CNN receives the output of the 2D TF representation.

[53] used VoiceLens model to detect numerous neurological problems simultaneously. It combines the capabilities of MFCCs with a two-phase multi-class classification module to develop an accurate voice-based disease prediction model. The first phase uses a stacked long short-term memory (LSTM) network to collect fine-grained information of these illnesses and their sequential variation patterns to detect baseline disease. In the second phase, a deep multilayer learnt descriptor analyses the discovered pathology samples to determine illness kinds. It used Saarbruecken Voice Database for the research. The model achieved 98.00% F1 score and 97.13% recall in the disease detection experiments, demonstrating its exceptional performance

## 3. Materials and Methods

The online available “Saarbruecken Voice Database” (SVD) published by the Institute of Phonetics of the University of Saarland is utilized for this research project, composed of vocal voices recorded from more than 2000 healthy and pathological subjects [54]. This data is a collection of vowels /a/, /i/, and /u/ and “Good Morning, how are you?” sentences, recorded with normal, low, high, rising, and falling pitch, available in both English and German languages. However, utilizing the /a/ vocalization subset of SVD remarks good classification results and is used in the literature [35, 55]. For our analysis, we have used the /a/ vowel phonation with a normal pitch in the English language. This subset comprised of 2,041 total sounds contributing 886 and 1,155 audio files from male and female subjects, respectively, (Figure 1), recorded at 50 kHz sampling rate with 16 bit-rate and at mono channel. In comparison, there are 259 and 428 healthy voices, 627 and 727 pathological voices of male and female, respectively, making a total of 687 healthy and 1,354 pathological voices (Figure 2). The overall statistics of the dataset are shown in Table 1.

Figures 3 and 4 reveal that the duration of the healthy voices varies in range 0.5 sec to 4.39 sec, while the pathological voices duration range in 0.3 sec to 2.63 sec making total duration of 687 sec and 1354 sec of healthy and pathological voices, respectively.

From the time and frequency domain plots shown below, it is clear that the amplitude lies within range -1 to 1 and most of the signal's energy lies in 70 dB to 80 dB. Figures 5 and 6 shows healthy voice plots for time domain and spectrogram, respectively.

Figures 7 and 8 shows voice pathology of both time domain and spectrogram plots.

### 3.1. Preprocessing

Machine learning (ML) and deep learning (DL) models require data in the form of vector representation of each sequence having the same length to perform matrix computation. The dataset that we have explored has a different duration range. In addition, from the statistics of the dataset, it is clear that there is a class imbalance of healthy and pathological voices. To overcome the above two defects, we adopt the sample padding and segmentation technique of signal processing, to keep all the voice's duration constant and to balance the samples at each class. Experimental results have shown that sample padding performs better than zero padding, in which the shorter signal is padded with its sample signal of the desired length. Since most of the voice signals have density higher than 1.5 sec. So, we have padded all the signals to 1.5 sec, especially for the signals that fall short. Further, for the signals which are greater than 1.5 sec are chuncked into segments. This is done to overcome the class imbalance. Figures 9 and 10 represent the statistics after padding and segmentation.

Due to the inherent complexity and a large number of layers in the deep learning model, they require a huge amount of data for training and better performance. Thus, we increase the number of samples by using the segmentation technique of signal processing. All the samples whose duration is greater than 1.5 sec are segmented into a different number of chunks based on the signal duration, while the last chunk is padded with its sample if its duration is less than 1.5 sec. After segmentation, we have now increased the number of samples in each class.

Table 2 shows the overall statistics of the data after segmentation. The number of healthy and pathological samples has now increased from 687 to 908 and 1,354 and 1,827, respectively. For our analysis and training DL model, we should have a balanced number of samples in each class. Based on the number of samples in the majority class (healthy), we have selected 908 (347 male and 561 female) samples from both healthy and pathological classes. The selected number of balance samples can visually be shown in Figure 11.

The time and frequency domain representations of chunked and padded signal from healthy and pathological classes are shown from Figures 12–15. From the figures, it can be seen that there is not any discontinuity after padding and segmentation in their time and frequency domains. So, we can use the data as originally recorded signals without any alteration for feature extraction and classification.

## 4. Proposed Methodology

### 4.1. Feature Extraction

To increase the performance of the classification model in terms of results (generalization) and computation time (speed of learning), feature extraction techniques are used to get the hidden patterns in the signal and to reduce the amount of redundant data from the dataset. Therefore, acceptable classification is derived from excellent and quality features. In Mel-frequency cepstral coefficients (MFCCs), features are commonly used in the literature for speech and sound processing. MFCCs computation is the replication of the human hearing system.

The MFCCs are extracted by first taking the Fourier transform of the widowed (framed) signal to convert it into the frequency domain. Let us denote the time domain signal **s**(**n**). Then for **i** number of frames, we have **s**_**i**_(**n**), where **n** represents frame samples. Generally, 1 to 13 MFCCs are extracted from each frame. **s**_**i**_(**k**) is the notation of the signal after calculating the discrete Fourier transform (DFT). The DFT of the signal is taken as

(1) $$\begin{array}{c} s_{i}\left(k\right)=\overset{N}{\underset{n=1}{\sum }}s_{i}\left(n\right)h\left(n\right)e^{-j2\pi kn/N}, \end{array}$$

where **h**(**n**) is an *N* sample long analysis window and *K* is the length of the DFT. The resulted power spectrum of each frame **s**_**i**_(**n**) is given as

(2) $$\begin{array}{c} \;P_{i}\left(k\right)=\frac{1}{N}{\left|s_{i}\left(k\right)\right|}^{2}. \end{array}$$

Then map the derived power of spectrum on the nonlinear Mel-scale followed by taking the logs of the power at each Mel-frequency and finally taking the discrete cosine transform of all the Mel-log powers. The amplitude of the resulting spectrum is the MFCCs. For our analysis, we have set the number of FFT to 2048, hop length to 512, and segment each signal into 0.5 sec to extract 13 MFCCs from each segmented sample of the signal at 50 kHz sampling rate. We have again segmented the voices so that we may have enough data for the deep learning model. Now we have 5,448 data samples.

The extracted MFCCs coefficients and the data from healthy and pathological voices are shown in Figures 16 and 17. Two different models are used to compare the results for the detection and classification of pathology in the voice signal and to compare the impact of the model trained on handcrafted extracted features and features extracted by the model itself. The first one is based on training 1D CNN on raw data, and the second one is based on training 2D CNN on the extracted MFCCs features. The voice signal is first padded to the 1.5-sec duration if duration falls short and segmented into 1.5 sec chunks if duration finds greater, using the sample padding and segmentation techniques of signal processing. The data is then framed and gets the 13 MFCCs from each frame to train 2D CNN. Used 70%, 10%, and 20% of train, validation, and test sets, respectively, of both the raw data and MFCCs features.  Figure 18 shows the proposed methodology for the classification of voice pathology.

### 4.2. Architecture of Model

Convolutional neural network (CNN) is a deep neural network model based on taking the mathematical function convolution to perform generalization from the input data. The CNN model has a variety of layers. The input layer is used to feed the data to the model, whereas the convolutional layer is used to extract high and low features from the data. The max-pooling layer is used to summarize and reduce the feature map.

#### 4.2.1. 1D CNN Architecture

We have used 6 convolutional layers with *relu* activation function having kernel size of three and enabling the zero-padding followed by the dropout layer to overcome overfitting and to regularize the weights. The six max-pooling layers are used after each convolution layer to extract and reduce the feature map. The data is then flattened and output is taken from the fully connected hidden dense layer with two neurons and *softmax* activation function. The model was complied with *Adam* [56] optimizer having 0.0001 learning rate, *binary_cross_entropy* as the loss function, and considering the *accuracy* as the evaluation metric. Finally, the model was fitted with train and validation data over 200 *epochs* and *batch_size* of six.

#### 4.2.2. 2D CNN Architecture

We have used two convolutional layers with *relu* activation function followed by the max-pooling with 3 × 3 kernel and batch-normalization layers. The data is then flattened, and output is taken from the fully connected dense layer with two neurons and *sigmoid* activation function. The model was complied with *Adam* optimizer having 0.001 learning rate, *binary_cross_entropy* as the loss function, and considering the *accuracy* as the evaluation metric. Finally, the model was fitted with train and validation data over 200 *epochs* and *batch_size* of 16.

The detailed architecture of the used 1D and 2D CNN models is tabulated in Table 3.

### 4.3. Evaluation Metrics

In this work, we set the parameter to compare the performance of the trained model with the existing work in the literature. To evaluate the performance of the binary classification model, we use various metrics based on the matrix called “confusion matrix”.

The performance of such a model is commonly evaluated using the data in the matrix. Below Table 4 is the foundation for the evaluation of all binary classification; the acronyms are also explained after the table.

Positive in the above table represent the class of interest.

- True negative (TN): when the data is actually negative and the model predict as negative
- False positive (FP): when the data is actually negative and the model predict as positive
- False negative (FN): when the data is actually positive and the model predict as negative
- True positive (TP): when the data is actually positive and the model predict as positive too

Based on the above confusion matrix result, there are some metrics for the model's performance evaluation.

- Accuracy: the ratio of the true predication to the overall prediction as

(3) $$\begin{array}{c} Accuracy=\frac{\left(TP+TN\right)}{All\;Predictions}. \end{array}$$

(b) Sensitivity: the ratio of the true positive to the total number positive predicted by the model

(4) $$\begin{array}{c} Sensitivity=\frac{TP}{TP+FN}. \end{array}$$

(c) Specificity: the ratio of the true negative to the total number of negative predicted by the model as

(5) $$\begin{array}{c} Specificity=\frac{TN}{FP+TN}. \end{array}$$

(d) Precision: out of all predicted positive, how many are actually positive. It is calculated as

(6) $$\begin{array}{c} Precision=\frac{TP}{FP+TP}. \end{array}$$

(e) F1 score: it is widely used evaluation metric for classification, which is the weighted average of precision and sensitivity

(7) $$\begin{array}{c} F1\;Score=2*\frac{\left(Sensitivity*Precision\right)}{Sensitivity\;Precision}. \end{array}$$

## 5. Results and Discussion

This section explains the details of experimental results obtained by our proposed CNN architectures. The goal is to divide the voice samples into healthy and pathological categories. First, we apply the raw audio signal to the 1D CNN that has been built. On the SVD dataset, we used feature extraction for 2D CNN training. We have extracted 13 MFCC features and sent them into the 2D CNN. The proposed models were trained, validated, and tested in the Google Colab. Then based on the selected metrics, evaluation of both trained models was carried out. Following that, both trained models were evaluated using the metrics chosen.1D CNN trained on raw data achieves 96% accuracy on the training set while 78% on the validation set. On the other hand, the 2D CNN model trained on MFCCs features generated an accuracy of 95% on the training set while 88% on the validation set (Table 5).

The accuracy plots against epochs on the training and validation set of both trained models are shown in Figure 19 and Figure 20, respectively. The loss plot on training and validation set against epochs is shown in Figures 21 and 22, respectively.

In addition, the trained models were evaluated and analyzed using the test data.  Table 6 shows the results obtained when both models are tested. The highest classification performance is obtained with 1D CNN for all the considered metrics in the table. Furthermore, the resulting test confusion matrices of both trained models are also shown in Figures 23 and 24. The confusion matrices indicate that out of 237 samples, 2D CNN correctly predicted 208 as pathological. As a result, the pathological class earned a class-wise accuracy of 87.76%. We only tested 105 samples with 1D CNN because we used raw audio signal, giving in a 95.23% testing accuracy. In the healthy class, 1D CNN had an accuracy of 91.15%, whereas 2D CNN had an accuracy of 79.89%. *A*: accuracy; *P*: precision; SN: sensitivity; SP: specificity; *F*: F1 score; TP: true positive; FP: false positive; FN: false negative; TN: true negative; PPV: positive predicted value; NPV: negative predicted value.

This paper proposes a method for automatically determining whether a voice is healthy or has a change in quality due to a pathological condition. Automatic detection is required since these illnesses quickly spread, although it is often underestimated. Machine learning is making a substantial contribution to the early identification and detection of diseases in cardiology, pulmonology, liver tumor segmentation, and other areas of healthcare. As a result, machine learning could be used efficiently for automatically classifying and detecting abnormalities in a person's voice for early diagnosis in a computer or mobile healthcare system. The SVD dataset is used for this purpose in contrast to other publicly available datasets. It is the world's largest publicly available dataset for voice analysis, with healthy and pathological vocal tones recorded from male and female patients. One of the most significant advantages of SVD was that the healthy and diseased voices were captured in the same context, allowing the model to learn the specific properties that distinguish the two types of voices. Previous research on other datasets [7] found that due to the fluctuation in the recording environment, the model became overfitted to the recording environment's properties rather than the real attributes that distinguish the voice classes.

In [4], experiments are carried out on vowels /a/, /i/, and /u/ at normal pitch results best performance for binary classification while using the vowel /u/. However, we aimed to enhance the performance by using the vowel /a/in this work. Thus using vowel /a/ at normal pitch, the signal was analyzed in both time and frequency domains. These signals are padded and segmented to ensure uniformity and increase the number of samples. Now the amount of healthy and pathological voices has increased from 687 and 1354 to 908 and 1827, respectively. Then features are extracted from the preprocessed signal followed by training of the models. 1D CNN achieves the highest train accuracy of 96% and test accuracy of 93.11%, while 2D CNN achieves train and test accuracy of 95% and 84.17%, respectively. Figures 19–22 illustrate both model's accuracy and loss plots on train and validation data, revealing that 2D models converge satisfactorily to the model's optimal weights and there is a sign of overfitting on 1D CNN.  Table 6 lists the comprehensive parameters of both models on test data, such as accuracy, F1 score, and recall. The confusion matrices also indicate the superiority of 1D CNN over 2D CNN. The models are better at detecting pathological than healthy class. This could be due to a lack of healthy person samples in the database compared to the number of pathological patient samples, as seen in Tables 1 and 2.

### 5.1. Comparative Analysis

This research was also compared to other studies that used the same workflow (Table 7). The key benefit of this study is that it produced better accuracy using the vowel /a/ than prior studies that employed all of the vowels to train the model [57]. With the LPCCs parameter in the /u/ vowel in men, the CNN classifier attained the best accuracy, 82.69%. Additionally, by utilizing vowel /a/ produced at normal pitch, our proposed 1D and 2D CNNs outperform previous work [21, 26]. [21] optimized their accuracy by utilizing the support vector machine technique. [26] convolutional layers and recurrent long short-term memory (LSTM) layers were applied to the raw audio signal to achieve a 68.08% on test data. Our future research will expand on the current study, but we will limit the number of disorders studied to only those with the most samples, and we will train distinct models for males and females. We will see if practicing with vowel combinations like /a/, /i/, and /u/ can assist with accuracy. We will also use data from other publicly available datasets to overcome the disadvantages of using only the SVD database and to make the model suitable for deploying to the appliances for use in real-life applications.

## 6. Conclusions

This work proposed and implemented a system for pathological voice detection using deep learning methods. The recordings of the sustained vowel /a/ were used for training and testing because they prevent linguistic artifacts and are commonly used in voice evaluation applications. The pathological data were recorded at normal pitch and were from 687 healthy and 908 pathological participants. To maintain homogeneity and enhance the number of samples, these signals are padded and segmented. MFCCs features were retrieved from the preprocessed data to acquire voice information from these recordings. Two types of classifiers based on the following deep learning approaches were explored to develop the most optimal classification model: 1 D CNN and 2D CNN. One model was trained on raw data, while the other was trained on extracted characteristics. This work stands out in the literature because of the increased number of samples and the use of two pipelines to compare performance. The best train and test results come from a 1D CNN; however, it is overfitting when compared to a 2D CNN, which generalizes the data better and has lower train and validation loss. Based on the results, it can be concluded that the model trained on handcrafted features performs better for speech processing than the model extracting features itself. Finally, the suggested 2D CNN model for early detection of vocal pathology can be implemented on a computer or a mobile phone. To relate the data to real-world settings, the suggested model needs to be trained on data with some discontinuity. This work should also be expanded to multiclass classification and enhance the performance of 1D CNN on raw data by increasing the number of samples because it saves a lot of time by not having to create a feature vector.

## Figures and Tables

**Figure 1:** Gender base statistics.

**Figure 2:** Diagnosis base statistics.

**Figure 3:** Healthy duration range.

**Figure 4:** Pathological duration range.

**Figure 5:** Time domain plot of healthy voice.

**Figure 6:** Spectrogram of healthy voice.

**Figure 7:** Time-domain plot of pathological voice.

**Figure 8:** Spectrogram of pathological voice.

**Figure 9:** Gender base statistics after preprocessing.

**Figure 10:** Diagnosis base statistics after preprocessing.

**Figure 11:** Visual representation of selected samples.

**Figure 12:** Time-domain plot of healthy voice after padding.

**Figure 13:** Spectrogram plot of healthy voice after padding.

**Figure 14:** Time-domain plot of pathological voice after padding.

**Figure 15:** Spectrogram plot of pathological voice after padding.

**Figure 16:** Extracted MFCCs coefficients and data of healthy voice.

**Figure 17:** Extracted MFCCs coefficients and data of pathological voice.

**Figure 18:** Block diagram of the proposed methodology.

**Figure 19:** 1D CNN performance.

**Figure 20:** 1D CNN loss plot.

**Figure 21:** 2D CNN Performance.

**Figure 22:** 2D CNN loss plot.

**Figure 23:** 1D CNN confusion matrix.

**Figure 24:** 2D CNN confusion matrix.

**Table 1:** Dataset statistics.

Class	Healthy		Pathological	
Gender	Male	Female	Male	Female
No of voice samples	259	428	627	727
Total	687		1,354	

**Table 2:** Dataset statistics after segmentation.

Class	Healthy				Pathological			
Gender	Male		Female		Male		Female	
No. of voice samples	Before segmentation	After segmentation	Before segmentation	After segmentation	Before segmentation	After segmentation	Before segmentation	After segmentation
	259	347	428	561	627	840	727	987
Total	Before segmentation		After segmentation		Before segmentation		After segmentation	
	687		908		1,354		1,827	

**Table 3:** Experiments with different CNN architecture.

Experiment	Architecture of CNN models
1D CNN	Convolutional layers: 6
	[(512 × 3 × 3) + dropout(0.25) + maxpool(2 × 2), (128 × 3 × 3) + dropout(0.25) + maxpool(2 × 2), (128 × 3 × 3) + dropout(0.25) + maxpool(2 × 2), (64 × 3 × 3) + dropout(0.5) + maxpool(2 × 2), (32 × 3 × 3) + dropout(0.5) + maxpool(2 × 2), (16 × 3 × 3) + dropout(0.5) + maxpool(2 × 2)]
2D CNN	Convolutional layers: 2
	[(16 × 3 × 3) + maxpool(2x2) + batchnormalization, (32 × 3 × 3) + dropout(0.3) + maxpool(2 × 2) + batchnormalization]

**Table 4:** Confusion matrix.

	Predicted negative	Predicted positive
Actual negative	TN	FP
Actual positive	FN	TP

**Table 5:** Training and validation accuracy comparison.

Model	Training accuracy	Validation accuracy
1D CNN	96%	78%
2D CNN	95%	88%

**Table 6:** Comparative evaluation of CNN models.

Model	*A*	*P*	*F*	SP	SN	TP	FP	FN	TN	PPV	NPV
1D CNN	93.11%	93.22	93.12%	91.15%	95.23%	100	10	5	103	90.90%	95.37%
2D CNN	84.17%	84.19%	84.12%	79.89%	87.76%	208	40	29	159	83.87%	84.57%

**Table 7:** Comparative evaluation with previous works on the same dataset.

Work	Accuracy
[57]	82.69%
[21]	84%
[26]	68.08%
1D CNN (proposed)	93.11%
2D CNN (proposed)	84.17%

## Data Availability

The dataset used in this study is available at http://stimmdb.coli.uni-saarland.de/index.php4#target.
